The article "Effects of Apatinib Mesylate Monotherapy on the Incidence of Adverse Reactions and Immune Function in Patients with Breast Cancer after Radical Mastectomy" was retracted in 2023. Reasons: signs of a paper mill; compromised peer review; unreliable results or conclusions.

# Effects of Apatinib Mesylate Monotherapy on the Incidence of Adverse Reactions and Immune Function in Patients with Breast Cancer after Radical Mastectomy

**DOI:** 10.1155/2022/4022282

**Published:** 2022-08-10

**Authors:** Sen Lin, Meichun Zang

**Affiliations:** ^1^Department of General Surgery, People's Liberation Army Navy 971 Hospital, Qingdao, Shandong, China; ^2^Department of Obstetrics and Gynecology, People's Liberation Army Navy 971 Hospital, Qingdao, Shandong, China

## Abstract

**Objective:**

To assess the effects of monotherapy with apatinib mesylate on the incidence of adverse events and immune function in breast cancer patients after a radical mastectomy.

**Methods:**

Between December 2018 and August 2020, 90 patients with breast cancer scheduled for a radical mastectomy in People's Liberation Army Navy 971 Hospital were randomly recruited and assigned at a ratio of 1 : 1 to receive either conventional treatment (conventional group) or apatinib mesylate after radical mastectomy (study group). The primary endpoint was disease control rate (DCR), and the secondary endpoints were adverse events and the immune function of the patients.

**Results:**

Monotherapy with apatinib mesylate was associated with a higher DCR (86.67%) versus conventional postoperative treatment (42.23%). All patients in the study group had documented adverse events, including 2 (4.45%) cases of headache, 3 (6.67%) cases of dizziness, 9 (20.00%) cases of hypertension, 6 (13.34%) cases of hand-foot syndrome, 3 (6.67%) cases of thrombocytopenia, 1 (2.23%) case of tinnitus, 7 (15.56%) cases of fatigue, 2 (4.45%) cases of anemia, 2 (4.45%) cases of oral pain, and 10 (22.23%) cases of leukopenia. There were 23 cases of intermittent discontinuation due to adverse events during treatment, 15 cases of dose reduction, and 3 cases of discontinuation due to adverse events. The difference in preoperative and postoperative T-cell subsets and natural killer (NK) cells between the two groups did not come up to the statistical standard (*P* > 0.05). Monotherapy with apatinib mesylate resulted in significantly lower levels of CD4+, CD4+/CD8+, and NK cells and higher CD8+ levels versus conventional treatment at 1 week and 4 weeks postoperatively (*P* < 0.05).

**Conclusion:**

Apatinib mesylate monotherapy after radical mastectomy yields a high DCR, a lower incidence of adverse events, and improved immune recovery. Clinical trials are, however, required prior to clinical promotion.

## 1. Introduction

Breast cancer is a disease in which the epithelial cells of the breast proliferate uncontrollably under the action of various carcinogenic factors, and it is one of the common malignant tumors in women [1]. The incidence of breast cancer has been on the rise due to environmental factors and the increasing pressure of life, and cervical cancer and breast cancer are the two latent culprits of cancer death in women, which seriously jeopardizes the health and life safety of women [2, 3]. The exact cause of breast cancer is poorly understood, although many signalling pathways and genetics have been identified [4]. Surgery is the preferred clinical treatment, with radical mastectomy being a standard radical mastectomy involving the removal of the entire affected breast and a 5 cm width of skin around the cancerous tumour, the fatty tissue surrounding the breast, the large and small chest muscles and their fascia, and all fatty tissue and lymph nodes in the axilla and subclavian area. Longitudinal, transverse, or shuttle-shaped incisions are acceptable, but the skin is generally excised no less than 3 CM from the tumor margin, with the surgical range extending from the clavicle to the superior rectus abdominis, outward to the anterior border of the latissimus dorsi muscle, and inward to the parasternal or midline sternum. This treatment is dictated by the physiological anatomical basis of the breast [4, 5].

The article "Effects of Apatinib Mesylate Monotherapy on the Incidence of Adverse Reactions and Immune Function in Patients with Breast Cancer after Radical Mastectomy" was retracted in 2023. Reasons: signs of a paper mill; compromised peer review; unreliable results or conclusions.

Despite a progressive decline in breast cancer recurrence and mortality due to the constant advancement of treatment techniques and the comprehensive application of systemic therapies, recurrence, and metastasis of breast cancer are still frequently seen in many patients [6]. Currently, radical surgery is the protocol of choice for the treatment of breast cancer, and aggressive postoperative chemotherapy is essential to prevent tumor recurrence and metastasis. Apatinib mesylate is an oral antiangiogenic targeted drug that blocks VEGFR-2 to suppress the proliferation of vascular endothelial cells by reducing the activation of mitogenic protein kinase (MAPK) to achieve antitumor effects [7–9]. In addition, Traditional Chinese medicine (TCM) treatment can be used as an adjuvant treatment for breast cancer to reduce the side effects and adverse effects of radiotherapy, chemotherapy, and endocrine therapy, thereby regulating the immune function and physical condition of patients [10]. In TCM, the cause of breast cancer is an internal injury to emotions, phlegm and blood stasis, and deficiency of righteousness, with the corresponding treatment methods including soothing the liver and relieving stagnation, resolving phlegm and dissipating blood stasis, regulating qi and blood, and nourishing the liver and kidney [11]. At present, the main treatment for breast cancer in TCM is compound decoctions, such as Tiaoshen Gongjian Decoction, Zigen Muli Decoction, and Qiyi Decoction [12]. Qiyi Decoction is mainly composed of Astragalus, Radix Angelicae Sinensis, and Rhizoma Atractylodis Macrocephalae and is effective in tonifying Qi and nourishing blood, resolving blood stasis and removing toxins, as well as strengthening the spleen and soothing the liver [13]. In view of the lack of reports, the aim of this study was to assess the effect of monotherapy with Apatinib Mesylate on the incidence of adverse events and immune function after radical mastectomy in breast cancer patients with the aid of the TCM Qiyi Decoction.

The article "Effects of Apatinib Mesylate Monotherapy on the Incidence of Adverse Reactions and Immune Function in Patients with Breast Cancer after Radical Mastectomy" was retracted in 2023. Reasons: signs of a paper mill; compromised peer review; unreliable results or conclusions.

## 2. Materials and Methods

### 2.1. Baseline Data

Between December 2018 and August 2020, 90 breast cancer patients scheduled for radical mastectomy at People's Liberation Army Navy 971 Hospital were recruited and allocated to either the conventional group (*n* = 45) or the study group (*n* = 45) using the two-colour method. This study was approved for execution by the Ethics Committee (Approval No. 20180915). Patients and their families were informed and signed consent forms.

### 2.2. Inclusion and Exclusion Criteria

#### 2.2.1. Inclusion Criteria

- With a history of pathologically confirmed breast cancer [14]
- All treated with radical breast cancer
- Patients were informed of this study and provided written informed consent

#### 2.2.2. Exclusion Criteria

- With abnormalities in the liver, kidney function, blood, and urine
- With severe acute myocardial infarction and pulmonary heart disease
- With consciousness or combined with mental illness

### 2.3. Methods

Qiyi decoction comprised 60 g of Astragalus, 30 g of Codonopsis, 15 g of Yujin, 15 g of Angelica, 30 g of Eclipta, 20 g of Atractylodes, 15 g of Paeonia lactiflora, 10 g of Chonglou, 30 g of Salvia, 10 g of Coix Seed, and 60 g of Liao JIangshi. The above herbs were decocted with water and administered twice daily for both groups [12].

Patients in the conventional group were treated with conventional treatment after radical mastectomy: 1250 mg/m^2^ of Capecitabine (Jiangsu Hengrui Pharmaceutical Co., Ltd., State Drug Administration: H20133365) was administered orally, twice a day in the morning and evening, with the total daily dose controlled within 2500 mg/m^2^.

All patients in the study group were treated with apatinib mesylate monotherapy after radical mastectomy: referring to the recommendations of the National Comprehensive Cancer Network (NCCN) guidelines, all patients were administered orally 500 mg of apatinib mesylate (Jiangsu Hengrui Pharmaceutical Co., Ltd., State Drug Administration: H20140103) once a day, without co-administration with other antitumor drugs. The drug was discontinued until the progression of the disease or the development of adverse events due to intolerance.

The article "Effects of Apatinib Mesylate Monotherapy on the Incidence of Adverse Reactions and Immune Function in Patients with Breast Cancer after Radical Mastectomy" was retracted in 2023. Reasons: signs of a paper mill; compromised peer review; unreliable results or conclusions.

The blood pressure, blood routine, urine routine, and ECG of the patients were monitored, adverse events that occurred after drug administration were also recorded, and the short-term treatment efficacy was evaluated after 4 weeks of medication.

### 2.4. Outcome Measures

- Disease control rate (DCR): the DCR of the two groups was evaluated as per the Evaluation Criteria for Treatment Efficacy of Solid Tumors [15], which can be divided into partial remission, stable disease, and disease progression, and DCR = (partial remission cases + stable disease cases)/total number of cases × 100%.
- Adverse events including headache, dizziness, hypertension, and hand-foot syndrome during the treatment of patients in the study group were recorded.
- Immune function: 5 mL of fasting venous blood was collected before, 1 week after surgery and 4 weeks after surgery, respectively, and centrifuged at 3000r/min for 15 min to isolate the supernatant which was stored for assay. T-lymphocyte subsets and NK cells (monoclonal antibody from BD, USA) were determined by flow cytometry.

### 2.5. Statistical Analysis

GraphPad Prism 8 software was used for image rendering, and SPSS22.0 software was used for data analyses. The count data were expressed as (*n* (%)) and processed by the Chi-square test, and the measurement data were expressed as ($\bar{x}$ ± *s*) and processed using the *t*-test. Differences were considered statistically significant at *P* < 0.05.

## 3. Results

### 3.1. Baseline Data

The baseline features of the patients in the conventional group (aged 23–82 years, mean age 45.23 ± 3.79 years, 23 cases in TNM stage II, 22 cases in TNM stage III, 19 cases of undergraduate and above, 15 cases of high schools/junior colleges, 8 cases of junior high schools, and 3 cases of elementary schools and below in terms of education level) were comparable with those of the study group (aged 22–79 years, mean age 45.17 ± 4.02 years, 24 cases in TNM stage II, 21 cases in TNM stage III, 20 cases of undergraduate and above, 16 cases of high schools/junior colleges, 7 cases of junior high schools, and 2 cases of elementary schools and below in terms of education level) (*P* > 0.05) (Table 1).

### 3.2. Disease Control Rate

Monotherapy with apatinib mesylate was associated with a higher DCR (86.67%) versus conventional postoperative treatment (42.23%) (Table 2).

### 3.3. Adverse Events

All patients in the study group had documented adverse events, including 2 (4.45%) cases of headache, 3 (6.67%) cases of dizziness, 9 (20.00%) cases of hypertension, 6 (13.34%) cases of hand-foot syndrome, 3 (6.67%) cases of thrombocytopenia, 1 (2.23%) case of tinnitus, 7 (15.56%) cases of fatigue, 2 (4.45%) cases of anemia, 2 (4.45%) cases of oral pain, and 10 (22.23%) cases of leukopenia. There were 23 cases of intermittent discontinuation due to adverse events during treatment, 15 cases of dose reduction, and 3 cases of discontinuation due to adverse events (Table 3).

The article "Effects of Apatinib Mesylate Monotherapy on the Incidence of Adverse Reactions and Immune Function in Patients with Breast Cancer after Radical Mastectomy" was retracted in 2023. Reasons: signs of a paper mill; compromised peer review; unreliable results or conclusions.

### 3.4. Immune Function

No statistically significant difference was found in preoperative and postoperative T-cell subsets and natural killer (NK) cells between the two groups (*P* > 0.05). Monotherapy with apatinib mesylate resulted in significantly lower levels of CD4+, CD4+/CD8+, and NK cells and higher CD8+ levels versus conventional treatment at 1 week and 4 weeks postoperatively (*P* < 0.05). (Table 4).

## 4. Discussion

In recent years, the incidence of breast cancer has been increasing due to environmental factors and the increase in life stress, which poses a serious threat to women's health [16]. The exact etiology of breast cancer is still poorly understood [17]. Although radical mastectomy is effective in the removal of the tumor lesion, the recurrence or metastasis rate of breast cancer remains high, so aggressive postoperative chemotherapy is usually adopted as countermeasure [4, 18]. There exist a large number of abnormal blood vessels around the tumor for the nutrition supply of the tumor, and vascular endothelial growth factor (VEGF) is closely related to neovascularization [19]. Previous research has shown that apatinib, an independently developed anticancer drug in China, competitively binds to the tyrosine ATP-binding site in the receptor cell and exerts an inhibitory effect on tumor angiogenesis. It is an oral antiangiogenesis-targeting drug that blocks VEGFR-2, thereby reducing the activation of mitogenic protein kinase (MAPK) and plays an antitumor role in inhibiting the proliferation of vascular endothelial cells in a variety of solid malignancies [20–24].

Here, monotherapy with apatinib mesylate was associated with a higher DCR (86.67%) versus conventional postoperative treatment (42.23%). All patients in the study group had documented adverse events, including 2 (4.45%) cases of headache, 3 (6.67%) cases of dizziness, 9 (20.00%) cases of hypertension, 6 (13.34%) cases of hand-foot syndrome, 3 (6.67%) cases of thrombocytopenia, 1 (2.23%) case of tinnitus, 7 (15.56%) cases of fatigue, 2 (4.45%) cases of anemia, 2 (4.45%) cases of oral pain, and 10 (22.23%) cases of leukopenia. There were 23 cases of intermittent discontinuation due to adverse events during treatment, 15 cases of dose reduction, and 3 cases of discontinuation due to adverse events. In this study, although the lesions showed a mild tendency of enlargement during the short discontinuation of the drug, the efficacy was enhanced again after retreatment with apatinib. Therefore, in this study, patients who developed adverse events were given an exploratory dosing frequency of 1-2 d active interruption after every 5 d of continuous dosing. After the administration of symptomatic treatment, most of them were found to be tolerable and controllable, and the adverse reactions arising from the administration of the drug were significantly lower than those of other chemotherapeutic agents. The reason may be attributed to the occurrence of multidrug resistance (MDR) associated with the ATP-binding cassette protein (ABC) transporter on the cell membrane surface [19]. ABC protein family excretes chemotherapeutic drugs from cells, thus attenuating the cytotoxic effects of the drugs; apatinib can increase the accumulation of adriamycin and rhodamine 123 in breast cancer resistance protein (BCRP, ABCG2) high expression cells, thereby significantly increasing the cytotoxicity of ABCB1 and ABCG2 substrates, and also reverses MDR by downregulating ABCB1 or ABCG2 expression to reverse MDR and further enhance drug sensitivity in ABCB1 or ABCG2 high-expressing resistant cell lines, which is consistent with the results of the present study [25]. Thus, apatinib mesylate is considered an ideal clinical treatment for patients with breast cancer after radical mastectomy, with controlled adverse events, and shows great potential as an alternative after the failure of other chemotherapy regimens.

The article "Effects of Apatinib Mesylate Monotherapy on the Incidence of Adverse Reactions and Immune Function in Patients with Breast Cancer after Radical Mastectomy" was retracted in 2023. Reasons: signs of a paper mill; compromised peer review; unreliable results or conclusions.

It has been reported that cellular immunity is the main antitumor immunity, dominated by T-lymphocyte subsets, NK cells. CD4+ and CD8+ regulate the body's cellular immunity, and the T-lymphocyte subsets and cells of breast cancer patients are lower than those of the healthy population. Herein, no statistically significant difference was found in preoperative and postoperative T-cell subsets and natural killer (NK) cells between the two groups (*P* > 0.05). Monotherapy with apatinib mesylate resulted in significantly lower levels of CD4+, CD4+/CD8+, and NK cells and higher CD8+ levels versus conventional treatment at 1 week and 4 weeks postoperatively (*P* < 0.05). Prior studies found that a high CD8+ expression level suppresses the body's immune response, while a lower CD4+/CD8+ ratio indicates aggravation of the disease and poor prognosis [26]. NK cells are the most representative immune cells in the body's antitumor defense function with a broad-spectrum tumor cell killing function [27]. The results of the present study indicate that monotherapy with apatinib mesylate inhibits cellular immune function and better protects immune function, which is consistent with the results of previous studies.

The article "Effects of Apatinib Mesylate Monotherapy on the Incidence of Adverse Reactions and Immune Function in Patients with Breast Cancer after Radical Mastectomy" was retracted in 2023. Reasons: signs of a paper mill; compromised peer review; unreliable results or conclusions.

Apatinib mesylate can control tumor growth by blocking the blood supply of patients' tumors with promising therapeutic effects [21]. However, complications such as bleeding, perforation, rupture, and high blood pressure may occur during the administration of apatinib mesylate. To this end, traditional Chinese medicine was used herein as an adjuvant treatment [28]. Traditional Chinese medicine treatment is performed as per the characteristics of etiology and pathogenesis and the complexity of the disease, and syndrome differentiation and treatment were conducted [29]. The determinants of the disease are internal causes, and exogenous pathogens are the conditions for the onset. In TCM, breast cancer develops due to dysfunction of viscera, abnormal Qi and blood flow or congenital insufficiency, and depletion of viscera [30]. Thus, it is important to maintain the righteous qi and enhance the Qi of the spleen and stomach [31]. In addition to TCM decoctions with antitumour effects, external TCM treatments such as acupuncture, moxibustion, blood cupping, and external application of Chinese herbs are also available [32].

The limitations of this study are the unknown mechanism of TCM treatment and the absence of long-term follow-up, which will be conducted in future studies to provide more reliable data for breast cancer treatment.

## 5. Conclusion

Apatinib mesylate monotherapy after radical mastectomy is associated with high DCR, a lower incidence of adverse events in patients, and improved immune recovery. Clinical trials are, however, required prior to clinical promotion.

## Figures and Tables

**Table 1:** Comparison of baseline data ($\bar{x}$± *s*).

Groups	*n*	Age	Mean age	TNM stage		Education level			
				II	III	Undergraduate and above	High schools/junior colleges	Junior high schools	Elementary schools and below
Conventional group	45	23–82	45.23 ± 3.79	23	22	19	15	8	3
Study group	45	22–79	45.17 ± 4.02	24	21	20	16	7	2
*t*	—	—		—	—	—	—	—	—
*P*	—	—		—	—	—	—	—	—

**Table 2:** Comparison of disease control rate (%).

Groups	*n*	Partial remission	Stable disease	Progressive disease	Disease control rate
Conventional group	45	11	8	26	19 (42.23)
Study group	45	22	17	6	39 (86.67)
*X* ^2^	—	—	—	—	19.397
*P*	—	—	—	—	<0.001

**Table 3:** Comparison of adverse events (%).

Groups	*n*	Headache	Dizziness	Hypertension	Hand-foot syndrome	Thrombocytopenia
Study group	45	2 (4.45)	3 (6.67)	9 (20.00)	6 (13.34)	3 (6.67)

*Groups*	*n*	*Tinnitus*	*Fatigue*	*Anemia*	*Oral pain*	*Leukopenia*
Study group	45	1 (2.23)	7 (15.56)	2 (4.45)	2 (4.45)	10 (22.23)

**Table 4:** Comparison of T-cell subsets and NK cells ($\bar{x}$± *s*).

Groups	Timepoints	Conventional group (*n* = 45)	Study group (*n* = 45)	*t*	*P*
CD4^+^	Preoperatively	80.45 ± 5.28	80.39 ± 6.01	0.050	0.960
	1 week postoperatively	58.35 ± 5.12	69.13 ± 6.21	8.985	<0.001
	4 weeks postoperatively	69.88 ± 5.35	80.02 ± 5.98^*∗*^	8.477	<0.001

CD8^+^	Preoperatively	25.88 ± 3.63	25.92 ± 3.45	0.054	0.957
	1 week postoperatively	40.25 ± 3.02	35.13 ± 2.68	8.506	<0.001
	4 weeks postoperatively	35.12 ± 3.44	30.08 ± 3.18^*∗*^	7.217	<0.001

CD4^+^/CD8^+^	Preoperatively	1.86 ± 0.24	1.88 ± 0.17	0.456	0.650
	1 week postoperatively	0.88 ± 0.02	1.24 ± 0.17	14.108	<0.001
	4 weeks postoperatively	1.23 ± 0.28	1.72 ± 0.35^*∗*^	7.334	<0.001

NK	Preoperatively	18.24 ± 3.03	18.21 ± 3.14	0.046	0.963
	1 week postoperatively	12.24 ± 2.15	14.96 ± 2.14	6.015	<0.001
	4 weeks postoperatively	15.02 ± 2.16	18.08 ± 2.58^*∗*^	6.101	<0.001

*Note.* ^*∗*^ indicates no statistically significant differences at 4 weeks postoperatively (*P* > 0.05).

The article "Effects of Apatinib Mesylate Monotherapy on the Incidence of Adverse Reactions and Immune Function in Patients with Breast Cancer after Radical Mastectomy" was retracted in 2023. Reasons: signs of a paper mill; compromised peer review; unreliable results or conclusions.

## Data Availability

All data generated or analyzed during this study are included in this published article.
